The article "Age and gender-specific antibiotic resistance patterns among Bangladeshi patients with urinary tract infection caused by Escherichia coli" was retracted in 2025. Reasons: unreliable results or conclusions; lack of ethics approval or compliance.

# Age and gender-specific antibiotic resistance patterns among Bangladeshi patients with urinary tract infection caused by *Escherichia coli*

**DOI:** 10.1016/j.heliyon.2020.e04161

**Published:** 2020-06-08

**Authors:** Ahmed Hossain, Saeem Arafat Hossain, Aneeka Nawar Fatema, Abrar Wahab, Mohammad Morshad Alam, Md. Nazrul Islam, Mohammad Zakir Hossain, Gias U. Ahsan

**Affiliations:** a Department of Public Health, North South University, Dhaka, 1229, Bangladesh; b Center for Climate Change and Environmental Research, BRAC University, Dhaka, Bangladesh; c NSU Global Health Institute, Dhaka 1229, Bangladesh; d National Institute of Ophthalmology, Dhaka, Bangladesh; e Medinova Medical Services Ltd., Dhaka, Bangladesh

**Keywords:** Clinical research, Diagnostics, Infectious disease, Public health, Urology, Antibiotic resistance, *Escherichia coli*, Urinary tract infection, Primary health care, Bangladesh

## Abstract

**Background:**

In Bangladesh, treatment for urinary tract infection has become increasingly difficult due to antibiotic resistance. In addition, the prescription of age and gender-specific drugs is still far from being practiced in Bangladesh. We are examining trends of antibiotic resistance per age and gender in patients with urinary tract infection (UTI) caused by the most frequent agent, *Escherichia coli*.

**Methods:**

We determined the resistance of 1663 *E. coli* isolates obtained from urine cultures. A sensitivity study using the Kirby-Bauer method was carried out to identify the antibiotic resistance trends.

**Results:**

Imipenem with 1.9% resistance of all isolates found to be the lowest percentage of resistance. Meropenem (2.8%), amikacin (2.8%), colistin (2.9%), and nitrofurantoin (15.8%) showed low resistance percentages. The sensitivity analysis suggests that age and gender (area under curve = 0.67) should be taken into consideration to prescribe amikacin. The increasing odds ratios (OR) by age groups suggest that amikacin is a less effective agent for older patients with UTIs. Moreover, nitrofurantoin (OR = 1.45, 95% confidence interval (CI) = 1.07–1.95) and colistin (OR = 2.09, CI = 1.13–3.76) were less effective against isolates obtained from males compared to isolates obtained from females. Meropenem was effective against bacteria obtained from all age groups and genders. On the other hand, efficacy of imipenem was lower in isolates obtained from adults older than 40 years (OR: 0.44 for < = 18 years, OR = 0.47 for 19–40 years, OR = 0.86 for 41–60 years; reference: > = 61 years).

**Conclusion:**

In Bangladesh, meropenem, imipenem, amikacin, colistin, and nitrofurantoin are suitable therapeutic alternatives against urinary tract pathogens. Among the oral agents, amikacin, colistin, and nitrofurantoin should be prescribed, taking consideration of age and gender. These results will assist physicians in prescribing effective primary care antibiotics for UTI patients and encouraging the implementation of health policies for a safe prescription of antibiotics.

The article "Age and gender-specific antibiotic resistance patterns among Bangladeshi patients with urinary tract infection caused by Escherichia coli" was retracted in 2025. Reasons: unreliable results or conclusions; lack of ethics approval or compliance.

## 1 Introduction

Urinary tract infections (UTIs) are among clinical practice's most common and recurrent bacterial infections and account for one-third of all community-acquired or nosocomial infections [1]. Literature indicates that the burden of bacterial diseases in South Asia is rising, and so globally [2].

There are many bacteria that can cause UTIs, but the most common pathogen is *E. Coli* [1]. One of the most important advances in modern medicine was the discovery of antibiotics, but their availability and expanded use slowly lead to microbial resistance for patients [3]. From the literature, it appears that about 15% of all prescription antibiotics are used to treat UTI [4]. Around 20–50% of all the antibiotic treatments are estimated to be inappropriately indicated, resulting in an increased risk of side effects, increased cost of treatment, and increased resistance [5].

The prime step in the treatment of bacterial UTI is treating patients with an effective antibiotic. However, the selection of the appropriate antibiotic is a big concern when treatment is to be given in primary health care (PHC) before isolating the causative agent and performing the test of sensitivity. Wide-spectrum antibiotics are commonly indicated to treat UTIs when, instead, a narrow-spectrum antibiotic could have been sufficient for an effective treatment [6]. In this scenario, after “blanket” use of antibiotics, resistance to antibiotics has emerged as a major concern in the world in recent years [7, 8, 9].

Resistance to antibiotics is a critical and extremely important problem in Bangladesh, where the infectious disease burden is high. A recent study in the UK has shown that antibiotic prescribing in primary care is declining, but this is not the case in Bangladesh [10]. Many medical doctors in Bangladesh prescribe antibiotics based on symptoms of UTI without a diagnosis based on urine culture. In fact, culture facilities are not available in many rural parts of Bangladesh. This could lead to self-medication and excessive antibiotic use [11, 12]. Resistance to antibiotics in bacteria can change with time and geographic location [13, 14, 15]. In addition, an UTI is usually related to age and gender. Doctors also need to update their awareness of the status of locally circulating strains and their antibiotic resistance patterns so that patients can be handled correctly and effectively.

The article "Age and gender-specific antibiotic resistance patterns among Bangladeshi patients with urinary tract infection caused by Escherichia coli" was retracted in 2025. Reasons: unreliable results or conclusions; lack of ethics approval or compliance.

Due to age and gender, UTIs may exhibit different epidemiological and etiological properties [16]. Isolates obtained from male or female might have different resistance profiles. Selection of the antibiotic to be prescribed against UTIs needs the support of local and current data. Furthermore, the preventive practice of UTI is rarely examined by taking into account age and gender. This research, therefore, explores the age and gender-specific trends of resistance to antibiotics in *E. Coli* caused UTIs amongst the population of Bangladesh.

## 2 Methods

From November 2017 until August 2018, we performed a cross-sectional study following the STROBE guideline. The sensitivity to amikacin, cefixime, ciprofloxacin, cotrimoxazole, meropenem, ceftriaxone, cephalexin, imipenem, nalidixic acid, and nitrofurantoin was determined for 1663 *E. coli* isolates obtained from various outlets of Medinova Medical Services Limited (MMSL) in Bangladesh. The research included both the male and female UTI patients above six years of age. The doctor suggested urinary infection based on a clinical examination of the visited patients' signs and symptoms, and then they were referred to the MMSL for urine culture and sensitivity testing. A positive culture of urine confirmed UTI cases. Reports on Urine Culture and Sensitivity were obtained from the MMSL database. We've taken on the reported *E. coli* samples for the analysis. So, we did not take the patients' informed consent.

According to the National Committee for Clinical Laboratory Standards, the antibiotic susceptibility examination was formulated using the disc diffusion method (Kirby-Bauer Method) [17]. The antibiotics discs used in this study included: amikacin (30μg), cefixime (5μg), ciprofloxacin (5μg), cotrimoxazole (1.25μg + 23.75μg), meropenem (10μg), ceftriaxone (30μg), cephalexin (30μg), imipenem (10μg), nalidixic acid (30μg), and nitrofurantoin (300μg). Samples with colony counts < 10^5^ cfu/ml were omitted. Quality assurance has been strictly controlled by the Clinical and Laboratory Standards Institute (CLSI) according to the “Performance Standards for Antimicrobial Susceptibility Testing” (i.e., the CLSI M100-S24 manual) [17].

Before the research started, we took the ethical clearance from the North South University review committee. The privacy and confidentiality of data concerning the personal identity of UTI patients was strictly protected.

### 2.1 Statistical analysis

Data was analyzed using R 3.3.1. All categorical variables (presented as frequencies and percentages) were determined using descriptive statistics. For the microbial-resistance to each antibiotic, we designed logistic regression models. The findings are reported by the odds ratios (ORs) and confidence intervals and significance was assumed when p < 0.05. ROC curves were used to predict antibiotic resistance based on age and gender.

The article "Age and gender-specific antibiotic resistance patterns among Bangladeshi patients with urinary tract infection caused by Escherichia coli" was retracted in 2025. Reasons: unreliable results or conclusions; lack of ethics approval or compliance.

## 3 Results

In Table 1, a descriptive analysis of age and gender between UTI patients is presented. It shows that among the 1663 reports of UTI patients, 1285 (77.27%) were females. The subjects' average age was 43.87 years, with a standard deviation of 22.8 years (range 6–87 years). Diffusion tests results indicated high rates of bacterial resistance to antibiotics, including; amoxicillin (90.0%), nalidixic acid (78.7%), cephalexin (84.1%), cefixime (57.5%), ceftriaxone (51.2%) and cotrimoxazole (47.1%) (Figure 1). The antibiotics that found lower rates of resistance among the *E. coli* isolates were meropenem (2.8%), imipenem (1.9%), amikacin (2.8%), colistin (2.9%), and nitrofurantoin (15.8%).

**Table 1:** Distribution of the demographic variables of the respondents (n = 1663).

Gender	Age Group				Total
	≤18	19–40	41–60	≥61	
Male	93 (24.6)	67 (17.7)	96 (25.4)	122 (32.3)	378
Female	166 (12.9)	416 (32.4)	399 (31.1)	304 (23.7)	1285

**Figure 1:** Distribution of the overall proportions of resistance to antibiotics by *E. coli* isolates obtained from UTI cases in Bangladesh.

The distribution of microbial-resistance to antibiotics by the patient age groups is given in Table 2. Isolates obtained from older patients seemed to have high resistance to amikacin and nitrofurantoin. UTI patients within the age group less than or equal to 18 years were 71% less resistant to amikacin compared to the patients of the age group 60 + years (OR = 0.29, Confidence Interval (CI) = 0.084–0.763). In addition, isolates obtained from patients aged 19–40 years were 43% less resistant to nitrofurantoin relative to patients aged 60 + years (OR = 0.57, CI = 0.390–0.816). Colistin also offered better efficacy against isolates obtained from younger patients compared to the older ones (60 + years). Efficacy of the two intravenous drugs, meropenem and imipenem, was similar against isolates obtained from all age groups. The resistance to imipenem, however, decreases as the odds ratios rise to nearly one as the age increases.

**Table 2:** Distribution and odds ratio (OR) of microbial-resistance to antibiotics according to age groups of the respondents.

Drugs	Age groups	Resistant n (%)	OR (CI)	P value
Amikacin	≤18 years	4 (1.56)	0.29 (0.084–0.763)	**0.024**
	19–40 years	8 (1.66)	0.31 (0.127–0.672)	**0.005**
	41–60 years	12 (2.44)	0.46 (0.216–0.918)	**0.032**
	≥61 years	22 (5.2)	*Reference*	
Nitrofurantoin	≤18 years	40 (15.87)	0.79 (0.517–1.192)	0.268
	19–40 years	57 (11.9)	0.57 (0.390–0.816)	**0.002**
	41–60 years	86 (17.70)	0.90 (0.642–1.262)	0.542
	≥61 years	80 (19.28)	*Reference*	
Meropenem	≤18 years	6 (2.32)	0.61 (0.215–1.495)	*0.302*
	19–40 years	11 (2.29)	0.60 (0.268–1.295)	0.198
	41–60 years	13 (2.63)	0.69 (0.323–1.451)	0.330
	≥61 years	16 (3.76)	*Reference*	
Imipenem	≤18 years	3 (1.16)	0.44 (0.099–1.43)	*0.212*
	19–40 years	6 (1.24)	0.47 (0.162–1.255)	0.144
	41–60 years	11 (2.23)	0.86 (0.364–2.021)	0.721
	≥61 years	11 (2.59)	*Reference*	
Colistin	≤18 years	10 (3.88)	1.68 (0.679–4.143)	*0.255*
	19–40 years	15 (3.11)	1.33 (0.598–3.096)	0.487
	41–60 years	13 (2.63)	1.12 (0.488–2.654)	0.787
	≥61 years	10 (2.35)	*Reference*	

Bold indicates significant at 5% significance level.

The article "Age and gender-specific antibiotic resistance patterns among Bangladeshi patients with urinary tract infection caused by Escherichia coli" was retracted in 2025. Reasons: unreliable results or conclusions; lack of ethics approval or compliance.

It appears from Table 3 that gender has a significant effect on the resistance to amikacin, nitrofurantoin, and colistin. The results show that bacteria from males are 2.27 times more resistant to amikacin than isolates obtained from females (CI = 2.27, CI = 1.22–4.11). Besides, isolates obtained from males were 2.09 times more resistant to colistin (CI = 2.09, CI = 1.13–3.76) and 1.45 times more resistant to nitrofurantoin (OR = 1.45, CI = 1.07–1.95), compared to isolates obtained from females. Both meropenem and imipenem were found similarly effective against isolates obtained from males and females.

**Table 3:** Distribution and odds ratio (OR) of microbial-resistance to antibiotics according to the gender of the respondents.

Drugs	Category (Gender)	Resistant n (%)	OR (CI)	P value
Amikacin	Male	18 (4.83)	2.27 (1.22–4.11)	**0.008**
	Female	28 (2.19)	*Reference*	
Nitrofurantoin	Male	75 (20.27)	1.45 (1.07 - 1.95)	**0.0138**
	Female	188 (14.9)	*Reference*	
Meropenem	Male	13 (3.45)	1.35 (0.68–2.53)	0.366
	Female	33 (2.58)	*Reference*	
Imipenem	Male	10 (1.64)	0.62 (0.29–1.40)	0.222
	Female	21 (2.65)	*Reference*	
Colistin	Male	18 (4.76)	2.09 (1.13–3.76)	**0.015**
	Female	30 (2.34)	*Reference*	

Bold indicates significant at 5% significance level.

### 3.1 Sensitivity analysis

The highest area under the ROC curve (AUC) given in Figure 2 is the best classification by age and gender. It shows that the amikacin line has the highest AUC of 0.67, which means that amikacin should be recommended for the UTI patients by taking into account the age and gender. Both colistin (AUC = 0.59) and imipenem (AUC = 0.60) have considerable variation against isolates resistant concerning gender. Thus, both drugs should be administered considering gender. The drug meropenem (AUC = 0.55) performs well against bacteria regardless of age and gender, and nitrofurantoin (AUC = 0.57) performs well regardless of gender. The intravenous drug meropenem, therefore, offers excellent activity against *E. coli*, and the medication may be administered to UTI patients irrespective of their age and gender.

The article "Age and gender-specific antibiotic resistance patterns among Bangladeshi patients with urinary tract infection caused by Escherichia coli" was retracted in 2025. Reasons: unreliable results or conclusions; lack of ethics approval or compliance.

**Figure 2:** Receiver operating characteristic curves for the *efficacy of* five antibiotics against *E. coli* isolates obtained from UTI cases in Bangladesh.

## 4 Discussion

Our study shows the distribution of antibiotic resistance among *E. coli* isolates obtained from UTI cases in Bangladesh, considering age and gender of the patients. Meropenem and imipenem were the selection of antibiotic therapy showed the highest sensitivity percentages among the isolates. But, as they are administrated intravenously, a closer control is required. In addition, as they are more expensive, they are not commonly indicated for routine UTI treatment. Other studies show similar findings regarding meropenem and imipenem [18, 19, 20].

Cotrimoxazole has historically been the drug's first line, but currently, it has become immune to UTI patients [19]. A few antibiotics, such as nalidixic acid and ciprofloxacin, then thrived [21, 22]. In this research, however, we found very high microbial-resistance to nalidixic acid, ciprofloxacin, and also antibiotics of the third generation, such as cefixime and ceftriaxone. The resistance rate for cotrimoxazole in our sample has been found to be similar from Senegal, Spain, and Taiwan but is much lower than that observed in India about ten years ago [22, 23]. Previously, few studies found that *E. coli* isolates have high rates of resistance to nitrofurantoin [24, 25, 26]. The present study showed much greater resistance of *E. coli* isolates to cephalexin compared with the 2015 study in Sudan [19]. Related research in rural Bangladesh found a remarkably lower resistance of *E. coli* to cephalexin (33%), cefixime (23%), ciprofloxacin (21%), ceftriaxone (17%), nitrofurantoin (3%) and nalidixic acid (37%) [27]. Another study, carried out in 2013 among women living in shanty towns in Dhaka reported maximum susceptibility to ceftriaxone, which contradicted our findings [28].

Our results indicated that *E. coli* from UTI are mostly susceptible to amikacin, meropenem, colistin, and imipenem. Akram et al. found much higher bacterial-resistance to amikacin in 2007 (51%) but lower resistance to imipenem in India [23]. Imipenem, meropenem, and colistin have been some of the few effective antimicrobials used to treat infections in this decade [29]. Colistin was included in the list of critically essential antimicrobials by the World Health Organization (WHO). In another study in 2014, however, it was reported that the use of colistin could increase development of resistance due to chromosomal mutations [30].

The article "Age and gender-specific antibiotic resistance patterns among Bangladeshi patients with urinary tract infection caused by Escherichia coli" was retracted in 2025. Reasons: unreliable results or conclusions; lack of ethics approval or compliance.

Nitrofurantoin was the first highly effective and safe antibiotic prescribed for UTI, decades ago, several bacterial pathogens are becoming resistant to it over time [31]. The prevalence of resistance to nitrofurantoin varied over the years, according to a few different studies summarized by Akter *et al.* in 2013: 10% (1987), 18.5% (1990), 43.6% (2002), 3.2% (2009) and 73.7% (2013) [32]. However, after discontinuing its use, is becoming more commonly used, and so we have microbial-resistance to it by just 15.6%. Several studies have recorded low bacterial-resistance (0–5%) in most parts of the world, although nitrofurantoin has long been used [33, 34]. Nitrofurantoin seems to be particularly useful for UTI treatment because it is highly concentrated in the urine [35].

We observed that amikacin and nitrofurantoin were more effective against isolates obtained from people of 60 years of age than their younger counterparts when testing the antibiotics in four different age groups. In the elderly population, however, it is best to stop amikacin and nitrofurantoin while empirically treating urinary tract infection. A research carried out in London in 2008 reflected a similar scenario for nitrofurantoin, but we were unable to compare such values because they used 16 years to be their demarcation age [36]. Both the meropenem and imipenem are used for intravenous administration as injection. Nitrofurantoin is an oral drug capsule, though. Nitrofurantoin is, therefore, more widely prescribed to UTI patients in Bangladesh. Our findings suggest that nitrofurantoin is highly responsive to age and gender and should, therefore, be given to patients after a culture test. The results indicate isolates collected from young or old people may have different resistance profiles.

This research has many strengths. Our study is the first to highlight the antibiotic susceptibility/resistance patterns of *E. coli* isolates from UTI cases, considering age and gender differences. These results are important to physicians as basis for prescription of effective antibiotics for UTI patients, preventing the emergence of new antibiotic-resistant strains by incorrect indications. Limitations include the study's use of the antimicrobial susceptibility testing approach for disc-diffusion, which does not always have a reliable antimicrobial resistance profile. In addition, regional variations in the pattern of resistance were not noted in this paper. A multi-level analysis with several diagnostic centers from urban and rural areas will help assess the overall generalizability of our findings for the UTI patients as a whole in a future objective.

The article "Age and gender-specific antibiotic resistance patterns among Bangladeshi patients with urinary tract infection caused by Escherichia coli" was retracted in 2025. Reasons: unreliable results or conclusions; lack of ethics approval or compliance.

## 5 Conclusions

High resistance to nalidixic acid, ciprofloxacin, cephalexin, cefixime, and ceftriaxone was detected among *E. coli* obtained from UTI cases in Bangladesh. In contrast, it was found that oral drugs like amikacin, colistin, and nitrofurantoin would be effective. The most effective drugs were meropenem and imipenem, but caution must be practiced because of potential side effects. *E. coli* isolates obtained from elderly patients were more resistant to amikacin and nitrofurantoin. In addition, isolates obtained from males exhibited greater resistance to amikacin, colistin, and nitrofurantoin. This study will help health care practitioners in proper antibiotic selection.

## Declarations

### Author contribution statement

A. Hossain: Conceived and designed the experiments; Analyzed and interpreted the data; Contributed reagents, materials, analysis tools or data; Wrote the paper.

S.A. Hossain: Conceived and designed the experiments; Analyzed and interpreted the data.

A.N. Fatema: Conceived and designed the experiments; Wrote the paper.

A. Wahab, M.M. Alam, M.N. Islam, M.Z. Hossain, G.U.Ahsan: Performed the experiments; Wrote the paper.

### Funding statement

This research did not receive any specific grant from funding agencies in the public, commercial, or not-for-profit sectors.

### Competing interest statement

The authors declare no conflict of interest.

### Additional information

Data associated with this study has been deposited at http://individual.utoronto.ca/ahmed_3/index_files/data/data.html.
